The article "Efficacy Evaluation of 64-Slice Spiral Computed Tomography Images in Laparoscopic-Assisted Distal Gastrectomy for Gastric Cancer under the Reconstruction Algorithm" was published in 2022. Journal: Contrast Media Mol Imaging.

# Efficacy Evaluation of 64-Slice Spiral Computed Tomography Images in Laparoscopic-Assisted Distal Gastrectomy for Gastric Cancer under the Reconstruction Algorithm

**DOI:** 10.1155/2022/2464640

**Published:** 2022-05-31

**Authors:** Weiguang Yu, Xing Li, Hongbo Zhou, Yang Zhang, Zhiguo Sun

**Affiliations:** ^1^Department of General Surgery, Affiliated Hongqi Hospital of Mudanjiang Medical University, Mudanjiang 157011, Heilongjiang, China; ^2^Internal Medicine Oncology, Affiliated Hongqi Hospital of Mudanjiang Medical University, Mudanjiang 157011, Heilongjiang, China; ^3^Department of Anatomy, Mudanjiang Medical University, Mudanjiang 157011, Heilongjiang, China

## Abstract

This study was aimed to analyze the application value of the filtered back-projection (FBP) reconstruction algorithm of computed tomography (CT) images in laparoscopic-assisted distal gastrectomy. In this study, 56 patients with gastric cancer were selected as research subjects and randomly divided into the control group (CT-guided laparoscopic radical gastrectomy) and the observation group (CT-guided laparoscopic radical gastrectomy with the FBP reconstruction algorithm), with 28 patients in each group. Fourier transform and iterative reconstruction were introduced for comparison, and finally, the postoperative curative effect and adverse events were compared between the two groups. The results showed that the CT image quality score processed by the FBP reconstruction algorithm (4.31 ± 0.31) was significantly higher than that of the iterative reconstruction method (3.5 ± 0.29) and the Fourier transform method (3.97 ± 0.38) (*P* < 0.05). The incidences of postoperative wound infection and gastric motility disorder (5.88% and 8.16%, respectively) in the observation group were significantly lower than those in the control group (8.21% and 10.82%, respectively) (*P* < 0.05). The levels of serum interleukin-6 (IL-6) (280.35 ± 15.08 ng/L) and tumor necrosis factor-*α* (TNF-*α*) (144.32 ± 10.32 ng/L) in the observation group after the treatment were significantly lower than those in the control group, which were 399.71 ± 14.19 ng/L and 165.33 ± 10.08 ng/L, respectively (*P* < 0.05). In conclusion, the FBP reconstruction algorithm was better than other algorithms in the processing of gastric cancer CT images. The FBP reconstruction algorithm showed a good reconstruction effect on CT images of gastric cancer; CT images based on this algorithm helped to formulate targeted surgical treatment plans for gastric cancer, showing a high clinical application value.

## 1. Introduction

Gastric cancer is one of the most common malignant tumors in China, which has a serious impact on human health and even life. The 5-year survival rate of such malignant tumors is generally low; however, if it can be detected early and treated aggressively, the 5-year survival rate can reach more than 90%. Therefore, early detection, early diagnosis, and early treatment of this type of malignant tumor are very important [1, 2]. According to 2018 global survey data, the incidence and mortality of gastric cancer ranked fifth and second in malignant tumors, respectively, and showed an increasing trend with age [3, 4]. Early gastric cancer may not show obvious clinical symptoms. When the patient develops symptoms such as abdominal pain or discomfort, anemia, indigestion, dysphagia or obstruction, and other symptoms, it has mostly become advanced gastric cancer [5, 6]. At present, gastric cancer is mainly treated by surgery, and radiotherapy and chemotherapy are performed before and after surgery to enhance the curative effect [7]. Radical surgery is the main treatment for early gastric cancer; palliative surgery can be used when the tumor cannot be completely removed in advanced gastric cancer [8, 9]. The resection rate of early gastric cancer is high, up to 90%. Once in the advanced stage, the progression is rapid, and the complete resection rate is extremely low [10, 11]. In addition, doctors need to formulate corresponding treatment plans according to their special circumstances and choose the most suitable therapy for patients with different tumor stages, tumor types, and physical conditions [12, 13].

The article "Efficacy Evaluation of 64-Slice Spiral Computed Tomography Images in Laparoscopic-Assisted Distal Gastrectomy for Gastric Cancer under the Reconstruction Algorithm" was published in 2022. Journal: Contrast Media Mol Imaging.

With the continuous advancement of modern medical diagnosis technology, various types of medical equipment are also highly popularized, and various auxiliary inspection methods can be used in the medical field to take images, assist clinicians to determine the lesions of gastric cancer, and determine surgical planning [14, 15]. Among them, computed tomography (CT) imaging is an important means of gastric cancer detection, with high diagnostic accuracy and good adaptability. However, the current segmentation of conventional CT images has great limitations and challenges, and there are problems such as blurred lesion boundaries and insignificant differences in brightness [16, 17]. Image reconstruction technology plays an important role in many fields. Common CT image reconstruction algorithms include the Fourier transform method, the iterative reconstruction method, and the filtered back-projection (FBP) method. In the process of research and implementation of the FBP algorithm, there are a series of extremely complex image processing problems and mathematical calculation problems, which have the advantages of fast reconstruction speed and high image quality [18].

The article "Efficacy Evaluation of 64-Slice Spiral Computed Tomography Images in Laparoscopic-Assisted Distal Gastrectomy for Gastric Cancer under the Reconstruction Algorithm" was published in 2022. Journal: Contrast Media Mol Imaging.

At present, algorithms such as image reconstruction and computer-aided medical image analysis have obvious advantages in major breakthrough in technology and the improvement of medical level and have also become an effective way to solve problems in the medical image. Therefore, to solve blurred edges and insignificant differences in brightness of traditional CT images, a FBP reconstruction algorithm was introduced for image processing, and applied in laparoscopic-assisted radical gastrectomy to analyze its clinical application value.

## 2. Materials and Methods

### 2.1. Research Objects and Their Grouping

In this study, 56 patients with gastric cancer, admitted to the hospital from October 2019 to October 2020, were selected as research subjects, including 26 male patients and 30 female patients, aged 48–65 years old. Patients were randomly divided into a control group (CT-guided laparoscopic radical gastrectomy) and an observation group (64-slice spiral CT-guided laparoscopic radical gastrectomy with the FBP reconstruction algorithm), with 28 patients in each group. The average age of patients in the control group was 53.21 ± 7.28 years old, and the average age of patients in the experimental group was 54.08 ± 6.87 years old. This study had been approved by the ethics committee of hospital, and these patients and their families understood the research content and signed the informed consent.

Inclusion criteria were as follows: patients diagnosed with gastric cancer who underwent laparoscopic-guided radical gastrectomy for gastric cancer without restriction of pathological type; patients with complete case data; and patients with no radiotherapy or chemotherapy before surgery.

Exclusion criteria were as follows: patients with liver and kidney dysfunction or other system and organ diseases; patients with abnormal coagulation function and blood routine; and patients with other types of gastric diseases such as gastritis and gastric ulcer.

### 2.2. CT Scanning

Patients were scanned with 64-slice spiral CT. Patients were required to fast for 5 hours before the CT scan, but could drink a small amount of water for half an hour before the scan. Patients were in the supine position, and the scanning range was from the top of the diaphragm to the lower poles of both kidneys. Scanning parameters were defined as follows: tube voltage was 120 kV, tube current was 120 mAs, gantry rotation time was 0.6 seconds, detector collimation parameter was 65 × 0.618 mm, field of view was 340 mm × 340 mm, and matrix was 521 × 521.

The obtained CT-enhanced images were sent to the workstation for processing. All patients underwent contrast-enhanced CT scans of the abdomen. CT images were interpreted by two attending doctors or radiologists with rich clinical experience. If there was any dispute between two doctors or radiologists, they can consult with the third doctor or radiologist.

The article "Efficacy Evaluation of 64-Slice Spiral Computed Tomography Images in Laparoscopic-Assisted Distal Gastrectomy for Gastric Cancer under the Reconstruction Algorithm" was published in 2022. Journal: Contrast Media Mol Imaging.

### 2.3. Reconstruction of CT Images

The basis of CT image reconstruction was that the same X-ray intensity, passing through different substances, has different attenuations. Using this law, different substances in the human body can be distinguished.

The process of CT image reconstruction was described as follows. In simple terms, structures within each layer of the human body that were penetrated by X-rays in a CT scan can be divided into small cubes (called voxels: *Voxel*). Each small cube corresponded to a separate attenuation signal, which was input into the corresponding small grid (called pixel: *Pixel*) in the image plane matrix, and the attenuation signal of each voxel was input into the corresponding pixel. Then, it was reflected in different grayscale images, so as to realize the reconstruction of CT images. Figure 1 shows the flow of FBP reconstruction of CT images.

The central slice theorem of a two-dimensional image stated that the Fourier transform method *p*(*ϖ*) of the projection and *p*(*s*) of a two-dimensional function *f*(*x*, *y*) was equal to the slice of the function *f*(*x*, *y*) that passed through the origin in a direction parallel to the detector of the Fourier transform method *F*(*ϖx*, *ϖy*).

The one-dimensional continuous Fourier transform method pair is

(1) $$\begin{array}{c} F\left(W\right)=\int_{-\infty }^{+\infty }f\left(t\right)e^{-iWt}\text{d}t, \end{array}$$

(2) $$\begin{array}{c} f\left(t\right)=\frac{1}{2}\pi \int_{-\infty }^{+\infty }f\left(W\right)e^{-iWt}\text{d}W. \end{array}$$

The two-dimensional continuous Fourier transform method and the corresponding Fourier transform are given as follows:

(3) $$\begin{array}{c} F\left(\mu ,\nu \right)=\int_{-\infty }^{+\infty }\int_{-\infty }^{+\infty }F\left(t,z\right)e^{-j2\pi \left(\mu t,\nu z\right)}\text{d}t\text{d}z. \end{array}$$

The inverse transform is as follows:

(4) $$\begin{array}{c} f\left(t,z\right)=\int_{-\infty }^{+\infty }\int_{-\infty }^{+\infty }F\left(\mu ,\nu \right)e^{j2\pi \left(\mu t+\nu z\right)}\text{d}\mu \text{d}\nu . \end{array}$$

In the above equation, *f* is a two-dimensional function; (*μ*, *ν*) represents the two-dimensional Fourier transform of the function; and the Fourier transform of projection of each angle was a straight line passing through the center of the frequency domain coordinates and finally formed a point scattering shape. The density of original points of the central segment in the plane *ϖx* − *ϖy* was higher than that in the region farther from the origin, while the region near the origin of Fourier space was the low frequency region. Excessive weighting of low frequency components caused the image to become blurred. In order to eliminate the blurring effect, it should weight the Fourier space to make the density uniform. Therefore, a low frequency filter |*w*| was used to suppress low frequency components and improve the clarity of the image.

The article "Efficacy Evaluation of 64-Slice Spiral Computed Tomography Images in Laparoscopic-Assisted Distal Gastrectomy for Gastric Cancer under the Reconstruction Algorithm" was published in 2022. Journal: Contrast Media Mol Imaging.

The basic starting point of the R-L filter function was that the actual two-dimensional image function always had an upper frequency limit, so the filter function |*θ*| in frequency can be expressed as

(5) $$\begin{array}{c} H_{R-L}\left(\theta \right)=\left\{\begin{array}{c} \begin{array}{cc} \left|\theta \right|, & \left|\theta \right|\leq \theta_{0}, \end{array}\\ 0. \end{array}\right. \end{array}$$

Its filter function is shown in Figure 2.

Then, the continuous R-L convolution function is expressed in

(6) $$\begin{array}{c} H_{R-L}\left(R\right)=\theta_{0}^{2}\left[2\sin c\left(2\theta_{0}R\right)-\sin c^{2}\left(\theta_{0}R\right)\right]. \end{array}$$

The discretized R-L convolution function is shown in

(7) $$\begin{array}{c} H_{R-L}\left(nT\right)=\left\{\begin{array}{cc} \frac{1}{4T^{2}}, & n=0,\\ 0, & \text{even number}\left(n\right),\\ -\frac{1}{\pi^{2}n^{2}T^{2}}, & \text{odd number}\left(n\right). \end{array}\right. \end{array}$$

Different from the R-L filter function, the S-L filter function does not use a rectangular function to intercept the |*θ*| filter function in the frequency domain but uses some smoother window functions to constrain the filter function. The window function *W*(*θ*) is assumed as follows:

(8) $$\begin{array}{c} W\left(\theta \right)=\sin c\left(\frac{\theta }{2\theta_{0}}\right)\text{rect}\left(\frac{\theta }{2\theta_{0}}\right). \end{array}$$

Therefore, it could obtain that the S-L function could be expressed as follows:

(9) $$\begin{array}{c} H_{S-L}\left(\theta \right)=\left|\theta \right|\sin c\left(\frac{\theta }{2\theta_{0}}\right)\text{rect}\left(\frac{\theta }{2\theta_{0}}\right). \end{array}$$

The convolution function corresponding to the S-L filter function is expressed as follows:

(10) $$\begin{array}{c} H_{S-L}\left(R\right)=\frac{1}{2}{\left(\frac{2\theta_{0}}{\pi }\right)}^{2}\frac{1-4\theta_{0}R\sin\left(2\pi \theta_{0}R\right)}{1-{\left(4\theta_{0}R\right)}^{2}}. \end{array}$$

Its discretized convolution function is given as follows:

(11) $$\begin{array}{c} H_{S-L}\left(nT\right)=-\frac{2}{\pi^{2}T^{2}\left(4n^{2}-1\right)}. \end{array}$$

### 2.4. Evaluation Indicators

All patients included underwent contrast-enhanced abdominal CT scans before laparoscopic-assisted distal gastrectomy. CT images of patients in the observation group underwent FBP reconstruction, and the reconstruction effect was analyzed by comparing the image quality scores.

The article "Efficacy Evaluation of 64-Slice Spiral Computed Tomography Images in Laparoscopic-Assisted Distal Gastrectomy for Gastric Cancer under the Reconstruction Algorithm" was published in 2022. Journal: Contrast Media Mol Imaging.

Image quality was rated as follows: (1) the image quality was very poor, with blurred edges and large noise in structures such as the chest wall; (2) the image quality was poor, some artifacts were visible, and the diagnostic requirements cannot be met; (3) the image quality was general with low recognition; (4) the image quality was good with sharp edges; (5) the image quality was good with high recognition, and it can be used for diagnosis.

The incidence of adverse events and inflammatory response indexes of the two groups of patients were compared after surgery: serum interleukin-6 (IL-6) and tumor necrosis factor-*α* (TNF-*α*). Detection was completed according to the operation instructions of the IL-6 detection kit and the TNF-*α* detection kit, respectively.

### 2.5. Statistical Methods

SPSS 22.0 statistical software was used for data processing in this study. Measurement data were expressed as mean ± standard deviation (*x* ± *s*), and enumeration data were expressed as percentage (%). Pairwise comparisons were made using analysis of variance. The difference was statistically significant at *P* < 0.05.

## 3. Results

### 3.1. CT Manifestations of Gastric Cancer

Figure 3 shows CT images of 4 gastric cancer patients, including 2 male patients and 2 female patients, aged 52, 50, 50, and 54 years old, respectively. According to CT images of the four patients, the gastric wall of these patients was irregular or diffusely thickened, and the gastric cavity was deformed and narrowed. In addition, submucosal infiltration, thickening and sclerosis of the gastric wall, thick mucosal folds, and thinning or thickening of local blood vessels can be seen, and perigastric fat space appeared as a cord image.

### 3.2. The Reconstruction Effect of the CT Image Algorithm

To solve the noise and unclear image edges in conventional CT images under the premise of ensuring image quality, the initial image was reconstructed by introducing the Fourier transform method, the iterative reconstruction method, and the FBP reconstruction algorithm to compare the processing effects of different reconstruction algorithms on the image. The results are shown in Figure 4. CT reconstruction of different tumor node metastasis (TNM) stages of lung cancer suggested that CT images processed by the FBP reconstruction algorithm showed higher definition, clear edges, and no obvious noise.

### 3.3. Evaluation of Reconstruction Effect

Figure 5 shows the comparison results of CT images processed by the Fourier transform method, the iterative reconstruction method, and the FBP reconstruction algorithm, respectively.  Figure 5(a) shows the comparison of CT values of three algorithms with different tube currents. There was no statistically significant difference in CT values of three algorithms with different tube currents (*P* > 0.05), and there was no significant difference in CT values of three algorithms for the same tube current (*P* > 0.05). Figures 5(a) and 5(b) illustrate that the CT image quality score processed by the FBP reconstruction algorithm (4.31 ± 0.31) was significantly higher than that of the iterative reconstruction method (3.5 ± 0.29) and the Fourier transform method (3.97 ± 0.38) (*P* < 0.05). In addition, the CT image noise processed by the FBP reconstruction algorithm (5.28 ± 0.63) was significantly lower than that of the iterative reconstruction method (7.25 ± 0.59) and the Fourier transform method (18.97 ± 0.54) (*P* < 0.05).

The article "Efficacy Evaluation of 64-Slice Spiral Computed Tomography Images in Laparoscopic-Assisted Distal Gastrectomy for Gastric Cancer under the Reconstruction Algorithm" was published in 2022. Journal: Contrast Media Mol Imaging.

### 3.4. Postoperative Adverse Events in Patients

After two groups of patients were treated by laparoscopic-assisted distal gastrectomy under the guidance of different CT images, the results of postoperative adverse events were compared. As illustrated in Figure 6, the more common postoperative adverse events included wound infection, abdominal pain, nausea and vomiting, gastric motility disorder, and pulmonary disorders. The incidences of gastric motility disorder and wound infection were higher. The incidence of postoperative wound infection (8.21% vs. 10.82%) and gastric motility disorder (5.88% vs. 8.16%) in the observation group were significantly lower than that in the control group (*P* < 0.05).

### 3.5. Changes of Postoperative Inflammatory Response Indicators in Patients

Figure 7 shows the comparison of changes in the inflammatory response indexes IL-6 and TNF-*α* before and after the treatment in the control group and the observation group. It demonstrates that there was no significant difference in the levels of IL-6 and TNF-*α* between the two groups before the treatment (*P* > 0.05). The serum levels of IL-6 and TNF-*α* in the observation group after the treatment (280.35 ± 15.08 ng/L, 144.32 ± 10.32 ng/L) were significantly lower than those in the control group (399.71 ± 14.19 ng/L, 165.33 ± 10.08 ng/L) (*P* < 0.05).

## 4. Discussion

Gastric cancer can be divided into early gastric cancer and advanced gastric cancer. Its CT has various manifestations, such as early gastric cancer is difficult to detect on CT due to its small lesions, and gastroscopic examination is required for diagnosis at this time [19]. For advanced gastric cancer, the cancer has invaded the submucosal layer and even entered the muscularis. On CT, main manifestations are localized or diffuse gastric wall thickening, the gastric wall thickening is usually uneven, and even ulcers can be seen, and the localized appearance of this cancer is rigid [20, 21]. CT can not only show changes of the gastric wall itself but it can also show the tumor's invasion to the surrounding, local or distant metastasis, such as the perigastric lymph node enlargement, ascites, thickening of the omentum and mesentery, and implanted nodules, showing a high application value in the diagnosis and the treatment of gastric cancer [22, 23]. Gastric cancer is divided into four stages according to CT manifestations. Stage I: a mass confined to the gastric cavity without metastasis or invasion to adjacent organs; stage II: the thickening of the gastric wall greater than or equal to 1 cm; stage III: gastric cancer that has invaded adjacent organs in addition to local manifestations; and stage IV: distant metastasis. Therefore, gastric cancer can be diagnosed by staging based on CT findings and then help clinicians to formulate corresponding treatment plans, so that patients can receive the most suitable treatment [24, 25]. The filtered back-projection reconstruction algorithm is developed on the basis of the back-projection method, and the image sharpness is solved by adding a filter function.

The article "Efficacy Evaluation of 64-Slice Spiral Computed Tomography Images in Laparoscopic-Assisted Distal Gastrectomy for Gastric Cancer under the Reconstruction Algorithm" was published in 2022. Journal: Contrast Media Mol Imaging.

Tamura et al. [26] showed that the FBP reconstruction algorithm has fast reconstruction speed and high image quality and has become a commonly used CT image reconstruction method. CT images of gastric cancer patients were processed by introducing the Fourier transform method, the iterative reconstruction method, and the FBP reconstruction algorithm, respectively. The results showed that the CT image quality score processed by the FBP reconstruction algorithm was significantly higher than that processed by the iterative reconstruction method and the Fourier transform method (*P* < 0.05); and the CT image noise processed by the FBP reconstruction algorithm was significantly lower than that by the iterative reconstruction method and the Fourier transform method (*P* < 0.05). It is concluded that the FBP algorithm not only effectively solves the problems of large noise and unclear edges in conventional CT images but also its performance is significantly better than other algorithms. The research of Padole et al. [27] pointed out that although the iterative reconstruction algorithm was proposed earlier than filtered back-projection, it depended on the breakthrough of computer performance due to its huge computational load and slow reconstruction speed.

CT images reconstructed by the FBP algorithm were used for laparoscopic-assisted distal gastrectomy. The results showed that the incidence of postoperative surgical wound infection and gastric motility disorder in the observation group was significantly lower than that in the control group (*P* < 0.05). It may be because CT images reconstructed by the FBP algorithm better show stratification of lesions invading the gastric wall and make more accurate staging according to the degree of invasion, so as to formulate targeted treatment plans for patients, reducing the occurrence of various postoperative adverse events in patients [28, 29]. The levels of serum inflammatory response indexes IL-6 and TNF-*α* in the observation group after the treatment were significantly lower than those in the control group (*P* < 0.05). Similarly, reconstructed CT images helped doctors to better observe tumor metastasis in combination with images, make accurate staging diagnosis, and carry out corresponding treatment. Therefore, using it in laparoscopic-assisted distal gastrectomy for gastric cancer is of a high application value.

The article "Efficacy Evaluation of 64-Slice Spiral Computed Tomography Images in Laparoscopic-Assisted Distal Gastrectomy for Gastric Cancer under the Reconstruction Algorithm" was published in 2022. Journal: Contrast Media Mol Imaging.

## 5. Conclusion

The results of this study found that the FBP reconstruction algorithm showed better reconstruction effect on CT images of gastric cancer; CT images based on the algorithm were helpful to formulate targeted surgical treatment plans for gastric cancer, showing a high clinical application value. However, this study only performed CT scan diagnosis and image reconstruction analysis for patients with advanced gastric cancer, and the sample sources were concentrated and lacked representativeness. Therefore, in the follow-up research, it would improve and optimize this aspect, and further analyze the reconstruction algorithm of CT images and its application value in the diagnosis and treatment of malignant tumors. In conclusion, this study could provide a reference for the early diagnosis and treatment of gastric cancer and other diseases.

## Figures and Tables

**Figure 1:** The flow of FBP reconstruction of CT images.

**Figure 2:** R-L filter function.

**Figure 3:** CT findings of four gastric cancer patients. The red marked area in the figure indicates irregular or diffuse thickening.

**Figure 4:** Processing effects of different algorithms. T3 and T4 represent different TNM stages. The red marked area in the figure indicates irregular or diffuse thickening.

**Figure 5:** Evaluation of CT image reconstruction effect. (a) CT value. (b) Comparison of the image quality score. (c) Comparison of the image noise. *∗* meant significant difference compared with the Fourier transform method (*P* < 0.05) and # meant significant difference compared to the iterative reconstruction method (*P* < 0.05).

The article "Efficacy Evaluation of 64-Slice Spiral Computed Tomography Images in Laparoscopic-Assisted Distal Gastrectomy for Gastric Cancer under the Reconstruction Algorithm" was published in 2022. Journal: Contrast Media Mol Imaging.

**Figure 6:** The incidence of postoperative adverse events in patients. (a–g) Postoperative wound infection, pulmonary infection, abdominal infection, severe abdominal pain, nausea and vomiting, gastric motility disorder, and other complications, respectively. *∗* indicates the difference was significant compared with the control group (*P* < 0.05).

**Figure 7:** Comparison of inflammatory response indicators in patients: (a) comparison of the changes of IL-6 and (b) comparison of the changes of TNF-*α*. *∗* indicates a significant difference compared with the control group (*P* < 0.05).

## Data Availability

The data used to support the findings of this study are available from the corresponding author upon request.
